The article "LncRNA MNX1-AS1 drives aggressive laryngeal squamous cell carcinoma progression and serves as a ceRNA to target FoxM1 by sponging microRNA-370" was published in 2021. Journal: Aging (Albany NY).

# LncRNA MNX1-AS1 drives aggressive laryngeal squamous cell carcinoma progression and serves as a ceRNA to target FoxM1 by sponging microRNA-370

**DOI:** 10.18632/aging.202746

**Published:** 2021-03-19

**Authors:** Xiangyan Cui, Hong Yu, Tingting Yu, Dong Xiao, Xin Wang

**Affiliations:** 1 Department of Otolaryngology-Head and Neck Surgery, The First Hospital of Jilin University, Changchun 130021, China

**Keywords:** laryngeal squamous cell carcinoma, MNX1-AS1, miR-370, FoxM1

## Abstract

Long non-coding RNA (LncRNA) MNX1 antisense RNA 1(MNX1-AS1) is associated with the pathology of numerous cancers. But, the role and underlying pathways of MNX1-AS1 in the regulation of laryngeal squamous cell carcinoma (LSCC) is not known. We demonstrated remarkably elevated levels of MNX1-AS1 in the LSCC tissues, which was correlated with poor disease prognosis. Moreover, MNX1-AS1-silencing strongly suppressed LSCC cell proliferation, migration, and invasion. We also demonstrated that MNX1-AS1 sequesters that activity of miR-370, thereby releasing Forkhead Box ml (FoxM1) from the inhibitory actions of MNX1-AS1. Furthermore, the positive correlation of MNX1-AS1 and FoxM1 as well as the converse correlation between miR-370 and MNX1-AS1 (or FoxM1) were revealed in LSCC tissues using experiments. Based on rescue assays, FoxM1 overexpression or miR-370 downregulation partially recovered the inhibitory effect of MNX1-AS1 silencing on LSCC cells. Moreover, knockdown of MNX1-AS1 retarded tumor growth in nude mice model. In summary, these findings verified that MNX1-AS1 modulated LSCC progression by competitively binding with miR-370 to regulate FoxM1.

## INTRODUCTION

Laryngeal squamous cell carcinoma (LSCC) is a highly prevalent form of laryngeal cancers that has been rising worldwide in recent years [1]. Although much advancements have been made in multimodal therapy like surgical resection, chemotherapy, radiotherapy, and combined therapies, the 5-year overall survival (OS) rate of LSCC patients have not altered significantly due to late diagnosis and high propensity for metastasis [2, 3]. As such, it is urgent and crucial to explore novel prognosis markers and therapeutic targets for LSCC.

Long non-coding RNAs (lncRNAs) are >200 nucleotides (nt) long RNAs that do not code for proteins and are associated with numerous forms of cancers via its regulation of chromatin remodeling, transcriptional modulation, and post-transcriptional control [4, 5]. Multiple studies report involvement of lncRNAs in LSCC progression and function as tumor suppressors or oncogenes [6, 7]. For instance, LncRNA DLX6-AS1 contributes to the LSCC growth via the regulation of miR-376c [8]. Similarly, lncRNA XIST modulates the miR-144/IRS1 axis to accelerate LSCC progression [9]. Furthermore, LncRNA CDKN2B-AS1 serves as an oncogene in the pathogenesis of LSCC and work via sponging of miR-497 to upregulate CDK6 [10]. Alternately, LncRNA GAS5 functions as a tumor suppressor that inhibits LSCC progression by sponging miR-21 [11]. These studies implied that lncRNAs might act as novel targets for diagnosis and treatment of LSCC. LncRNA MNX1-AS1 was first implicated in the progression of ovarian cancer [12]. Accumulating evidence demonstrated that MNX1-AS1 played an oncogenic role in multiple malignancies including gastric cancer [13], esophageal squamous cell carcinoma [14], osteosarcoma [15], non-small cell lung cancer [16], hepatocellular carcinoma [17], prostate cancer [18], breast cancer [19] and cervical cancer [20] and so on. Although one study reported increased MNX1-AS1 expression in LSCC tissues based on the Cancer Genome Atlas Database (TCGA) analysis [21], little is known about its role and regulation in the pathogenesis of LSCC.

In this study, we demonstrated elevated MNX1-AS1 levels in LSCC tissues, which closely related with advanced UICC stage, lymph node metastasis, and poor prognosis. Additionally, using both *in vitro* and *in vivo* experimentation, we revealed MNX1-AS1 silencing reduced LSCC growth and metastasis by targeting the miR-370/FoxM1 pathway. Hence, this study established a new regulatory pathway of MNX1-AS1/miR-370/FoxM1 axis that modulates LSCC progression.

## RESULTS

### LSCC tissues had elevated MNX1-AS1 expression, which closely correlated with poor prognosis

To establish MNX1-AS1 levels in LSCC, we examined MNX1-AS1 levels in LSCC tissues and adjoining healthy tissue (ANT) samples. As illustrated in Figure 1A, MNX1-AS1 was augmented in LSCC tissues, relative to ANT. Next, using the average MNX1-AS1 level in LSCC tissues as a cut off, 40 LSCC patients were categorized as either high expressing or low expressing for subsequent Kaplan-Meier analysis. We showed that patients with high expression of MNX1-AS1 had advanced UICC stage, lymph node metastasis, and poor overall survival (OS) ratio, relative to patients with low expression of MNX1-AS1 (Table 1, Figure 1B).

**Table 1:** Association of MNX1-AS1 expression with clinicopathologic factors in 40 cases of patients with LSCC.

**Variables**	**No. of cases**	**MNX1-AS1 expression**		***p* value^a^**
		**High**	**Low**	
Age (years)				*p *= 0.5121
<60	24	13	11	
≥60	16	11	5	
Gender				*p *= 0.2046
Male	25	17	8	
Female	15	7	8	
UICC stage				***p *= 0.0315**
I-II	30	15	15	
III-IV	10	9	1	
Histological differentiation				*p *= 0.1140
Well and moderately	32	17	15	
Poor	8	7	1	
Lymph node metastasis				***p = *0.0060**
No	31	15	16	
Yes	9	9	0	

**Figure 1:** **MNX1-AS1 was upregulated in LSCC and correlated with poor prognosis.** (**A**) Real-time PCR (qRT-PCR) analysis of MNX1-AS1 expression in 40 primary LSCC tissues and matched adjacent normal tissues. (**B**) Kaplan-Meier survival curve indicated the high expression of MNX1-AS1 is associated with low survival rates. The median value of MNX1-AS1 expression levels in these LSCC tissues was used to stratify the high and low expression levels of MNX1-AS1. ^*^P < 0.05; ^**^P < 0.01.

### MNX1-AS1 knockdown inhibits LSCC growth in cell culture and nude mice

MNX1-AS1 levels were assessed in a LSCC cell line TU212 and in normal bronchial epithelial cell line (16HBE). As depicted in Figure 2A, MNX1-AS1 was strongly expressed in TU212 cells, as opposed to 16HBE cells. To elucidate the role of MNX1-AS1 in LSCC, we silenced MNX1-AS1 levels in TU212 cells, using sh-MNX1-AS1 (Figure 2B). CCK8 assay showed that MNX1-AS1 silencing severely inhibited LSCC cell proliferation in TU212 cells, as opposed to sh-NCs (Figure 2C). Moreover, colony forming assays confirmed that reduced number of colonies in the MNX1-AS1 silenced cells, relative to sh-NCs (Figure 2D). To ascertain the effect of MNX1-AS1 silencing on LSCC tumor growth in mice, we administered MNX1-AS1 silenced cells to nude mice and demonstrated significantly smaller tumor volume and weight in the TU212-sh-MMNX1-AS1 mice, as compared to the sh-NCs (Figure 2E–2F). IHC assay showed that the positive cells of Ki-67 were greatly reduced in sh-MNX1-AS1 group verses the sh-NC group (Figure 2G). Based on these data, MNX1-AS1 knockdown significantly decreased tumor growth in cell culture and in nude mice.

**Figure 2:** **Knockdown of MNX1-AS1 inhibits LSCC growth *in vitro* and *in vivo*.** (**A**) qRT-PCR analysis of MNX1-AS1 expression in human LSCC cell line TU-212 and normal bronchial epithelial cell line (16HBE). (**B**) qRT-PCR analysis of MNX1-AS1 expression in TU212 cells transfected with sh-NC and sh-MNX1-AS1. (**C, D**) cell proliferation and colony formation were determined in TU212 cells transfected with sh-NC and sh-MNX1-AS1. (**E–F**) The volume and weight of tumor from nude mice model were measured. (**G**) IHC assay was used to evaluate the protein expression of Ki-67 in tumor. ^*^P < 0.05; ^**^P < 0.01.

### Knockdown of MNX1-AS1 inhibits LSCC cell migration and invasion

Using wound healing and transwell invasion assays, we measured the impact of MNX1-AS1 depletion on LSCC migration and invasion abilities. We observed that MNX1-AS1 depletion suppressed TU212 cell migration and invasion (Figure 3A and 3B).

**Figure 3:** **Knockdown of MNX1-AS1 inhibits LSCC cell migration and invasion.** (**A**) Wound healing analysis of cell migration in TU212 cells transfected with sh-NC and sh-MNX1-AS1. (**B**) Transwell invasion analysis of cell invasion in TU212 cells transfected with sh-NC and sh-MNX1-AS1. ^*^P < 0.05; ^**^P < 0.01.

### MNX1-AS1 sponges miR-370 in LSCC cells

Cytoplasmic lncRNAs exerted their function through serving as competing endogenous RNAs (ceRNAs) to sequester miRNAs [22, 23]. To further examine the underlying pathways within the MNX1-AS1 network regulating LSCC, we evaluated the subcellular localization of in TU212 cells, and found MNX1-AS1 to be a primarily cytoplasmic lncRNA (Figure 4A). Thus, we select the miRNAs that bind with MNX1-AS1 using online software (LncBook, https://bigd.big.ac.cn/lncbook/index). Based on the bioinformatics analysis, we discovered that MNX1-AS1 shares sequence homology with miR-370 (Figure 4B). Luciferase reporter assay demonstrated that high-expressing-miR-370-TU212 cells obviously lowered WT-MNX1-AS1 luciferase activity of, not but of MT-MNX1-AS1 (Figure 4C). To further confirm the physical interaction between MNX1-AS1 and miR-370, RNA-Pull down assays were carried out in TU212 cells, and revealed that MNX1-AS1 was pulled down by Bio-wt- miR-370, while miR-370-mut could not pull down MNX1-AS1 (Figure 4D). Moreover, using qRT-PCR, we demonstrated that miR-370 levels are significantly upregulated in MNX1-AS1-depleted TU212 cells (Figure 4E), whereas miR-370 upregulation or downregualtion did not change MNX1-AS1 levels in TU212 cells (Figure 4F). Additionally, we revealed very low levels of miR-370 in LSCC tissues and cell lines (Figure 4G and 4H). Moreover, there existed a negative relationship between miR-370 and MNAX1-AS1 levels in LSCC tissues (Figure 4I). Based on these data, miR-370 may be a downstream target of MNX1-AS1 in LSCC cells.

**Figure 4:** **MNX1-AS1 sponges miR-370.** (**A**) The MNX1-AS1 expression was examined in cytoplasm and nucleus of TU212 cells. U6 was used as the nuclear control and GAPDH was used as the cytoplasmic control. (**B**) The predicted miR-370 binding sites in the region of MNX1-AS1 and the corresponding mutant sequence were shown. (**C**) Effect of miR-370 on the luciferase activity of WT-MNX1-AS1 and MT-MNX1-AS1 reporter systems was detected via luciferase reporter assay. (**D**) RNA-Pull down assay was conducted to assess the relationship between miR-370 and MNX1-AS1. (**E**) The expression of miR-370 was examined in TU212 cells transfected with sh-MNX1-AS1 or sh-NC. (**F**) MNX1-AS1 expression was examined by qRT-PCR in TU212 cells transfected with miR-370 mimics, miR-NC, miR-370 inhibitor (anti-miR-370) and anti-miR-NC. (**G**) The expression of miR-370 was examined in LSCC tissues and adjacent normal tissues. (**H**) qRT-PCR analysis of the expression of miR-370 in human LSCC cell line TU-212 and normal bronchial epithelial cell line (16HBE). (**I**) Correlation between MNX1-AS1 and miR-370 expression in LSCC tissues was analyzed by Pearson’s correlation analysis. ^*^P < 0.05; ^**^P < 0.01.

### MNX1-AS1 serves an oncogenic role in LSCC via modulation of the miR-370/FOXM1 pathway

A previous study demonstrated that miR-370 inhibited LSCC tumorigenesis and development by targeting FoxM1 [24]. To assess a potential oncogenic role of MNX1-AS1 on LSCC via regulation of the miR-370/FoxM1 pathway, we examined the relationship between MNX1-AS1, miR-370, and FoxM1 in LSCC cells. We discovered that MNX1-AS1 silencing markedly suppressed FoxM1 levels in TU212 cells, whereas miR-370 inhibitor partially reverse this trend (Figure 5A and 5B). In addition, we revealed that FoxM1 levels increased in LSCC tissues (Figure 5C). Moreover, FoxM1 levels were negatively correlated with miR-370 (Figure 5D), and positively correlated with MNX1-AS1 (Figure 5E). Finally, we checked the effects of miR-370 and FoxM1 on MNX1-AS1 depleted-inhibited proliferation, colony formation, migration, and invasion. We found that miR-370 silencing or FoxM1 overexpression partially reversed the MNX1-AS1 silencing-mediated inhibitory effect in TU212 cells (Figure 5F–5I). These results determine convincingly that MNX1-AS1 regulates LSCC progression via miR-370/FoxM1 axis.

**Figure 5:** **MNX1-AS1 exerts tumor-promoting role in LSCC by regulating the miR-370/FoxM1 axis.** (**A, B**) The expression of FoxM1 on mRNA and protein levels was examined in TU212 cells transfected with sh-NC, sh-MNX1-AS1, and sh-MNX1-AS1+ anti-miR-370. (**C**) The mRNA expression of FoxM1 was examined in LSCC tissues and adjacent normal tissues. (**D**) Correlation between FoxM1 and miR-370 expression in LSCC tissues was analyzed by Pearson’s correlation analysis. (**E**) Correlation between MNX1-AS1 and FoxM1 expression in LSCC tissues was analyzed by Pearson’s correlation analysis. (**F–I**) Cell proliferation, colony formation, migration and invasion were detected in TU212 cells transfected with sh-NC, sh-MNX1-AS1, and sh-MNX1-AS1+ anti-miR-370 and sh-MNX1-AS1+FoxM1. ^*^P < 0.05; ^**^P < 0.01.

## DISCUSSION

Multiple reports confirmed that lncRNAs played a vital role in LSCC cell physiology and pathogenesis, and might act as diagnosis markers and therapy agents [6, 7]. Here, we aimed to clarify the precise role and uncover potential pathway of MNX1-AS1 regulation in LSCC. Here, we discovered that lncRNA MNX1-AS1 accelerated LSCC progression via miR-370/FoxM1 axis, indicating that MNX1-AS1 may be a potential therapy target for LSCC.

MNX1-AS1 was reported to serve as an oncogenic lncRNA in numerous forms of cancers [12–20]. For instance, MNX1-AS1 overexpression promotes gastric cancer progression via the EZH2/BTG2 and miR-6785-5p/BCL2 axis [13]. MNX1-AS1 contributed to bladder cancer initiation and progression via the modulation of miR-218-5p/RAB1A pathway [25]. MNX1-AS1 drove lung cancer growth and metastasis using the miR-527/BRF2 pathway [26]. Here, we discovered MNX1-AS1 levels to be up-regulated in LSCC tissues, which further confirmed the previous result from TCGA [21]. In addition, increased MNX1-AS1 was closely correlated with advanced UICC stage, lymph node metastasis and short survival of patients with LSCC. Subsequent loss-of-function assays revealed that MNX1-AS1 depletion reduced LSCC growth and metastasis *in vitro*, as well as inhibited tumorigenesis of LSCC *in vivo*. These data imply that MNX1-AS1 serves as an oncogene in LSCC.

A great evidence suggested that lncRNA can sequester miRNA and halt their suppression of miRNA-target genes [27]. MNX1-AS1 was reported to interact with multiple miRNAs within cancerous cells; namely, miR-218-5p [25], miR-34a [14], miR-527 [26], miR-6785-5p [13] and miR-4443 [28], indicating that MNX1-AS1 acts as a ceRNA to modulate tumorigenesis and progression. Here, we select miRNAs that can bind with MNX1-AS1 using LncBook online software. Among miRNAs, we chose to study miR-370 due to its essential role in cancer progression. miR-370 was shown to be downregulated and play a suppressive role in multiple cancers [29–31]. For LSCC, miR-370 expression was downregulated and function as a tumor suppressor in LSCC [24]. Through luciferase and RNA-Pull down assays, we further confirmed that miR-370 could bind with MNX1-AS1 in LSCC cells. Moreover, our results revealed that miR-370 levels were markedly elevated in MNX1-AS1-depleted TU212 cells. We also found that miR-370 levels were downregulated in LSCC tissues and cells. MNX1-AS1 levels were inversely associated with miR-370 levels in LSCC tissues. Moreover, miR-370 silencing partly rescued the inhibitory effects mediated by MNX1-AS1 depletion in LSCC cells. Based on these data, MNX1-AS1 modulated LSCC progression by acting as a ceRNA by sponging miR-370.

Forkhead box M1 (FoxM1) is a well established downstream target of miR-370 in LSCC [24]. FoxM1, belonging to the Fox transcription factor family, was related to tumor formation in multiple cancers [32, 33]. In LSCC, FoxM1 was shown to be elevated and served as a tumor promoting gene [34, 35]. Thus, we hypothesized that MNX1-AS1 modulates the miR-370/FoxM1 pathway in LSCC. Here, we discovered that FoxM1 expression was elevated in LSCC tissues, similar to what we demonstrated previously [34, 35]. In addition, the positive correlation of MNX1-AS1 and FoxM1 as well as the converse correlation between miR-370 and MNX1-AS1 (or FoxM1) were revealed in LSCC tissues. Of note, downregulation of miR-370 or upregulation of FOXM1 partially reversed the MNX1-AS1 silencing-mediated suppressive effects in TU212 cells. These findings indicate that MMX1-AS1 serves as an oncogene in LSCC by modulating miR-370/FoxM1 pathway.

In summary, we showed that MNX1-AS1 depletion retarded LSCC progression via miR-370/FoxM1 axis. Thus, MNX1-AS1 may be a promising new therapeutic target for LSCC. However, further studies are required to provide a deep understanding of the clinical translation of the MNX1-AS1/miR-370/FoxM1 axis in LSCC.

## MATERIALS AND METHODS

### Clinical samples

40 LSCC tissue samples and adjoining non-cancerous matched tissue samples were retrieved from patients undergoing partial or total laryngectomy between March 2014 and Mach 2015 at the First Hospital of Jilin University, under approval from Jilin University. All informed consents were signed by all patients. All patients did not receive any tumor treatment before admission. All tissues were flash-frozen in liquid nitrogen within 10 min of extraction and stored at −80°C until further examination.

### RNA purification and real-time quantitative PCR

Total RNA was extracted from cells or tissues with TRIzol reagent (Invitrogen, Carlsbad, CA) following manufacturer’s guidelines. The RNA was employed for the synthesis of cDNAs with Primescript RT reagent kit (Takara, Dalian, China). cDNAs were amplified and quantified by with SYBR Green mix (Takara) in Applied Biosystems 7500 instrument. Primer sequences used in this study were described previously [13, 24, 28]. Relative gene expression was measured by −2^ΔΔCt^ method. Internal controls were GAPDH and U6 for MNX1-AS1/FOXM1 and miR-370, respectively.

### Cell culture

Human LSCC cell line TU-212 and healthy bronchial epithelial cell line (16HBE) were bought from Shanghai Huiying Biological Technology (Shanghai, China), and maintained in Dulbecco’s modified Eagle’s Medium (DMEM) with 10% fetal bovine serum (FBS), 100 U/mL penicillin and 0.1 mg/mL streptomycin in a humid environment at 37°C with 5% CO2.

### Plasmids, mimics, inhibitor and plasmid incorporation

The plasmids used were as follows: shRNA against MNX1-AS1 (sh-MNX1-AS1) and negative control (NC) shRNA (sh-NC) in pLKO.1-puro vector (TransBio, Shanghai, China); miR-370 mimics, miR-370 inhibitor (anti-miR-370) and their NC (miR-NC or anti-miR-NC) (GenePharma, Shanghai, China). TU212 cells were incorporated with the indicated plasmid, namely, either mimic, inhibitor or shRNA with Lipofectamine^®^ 3000 (Invitrogen), following manufacturer’s guidelines. 2 × 10^5^ TU212 cells were plated and incorporated with pLKO.1-puro-sh-MNX1-AS1 or pLKO.1-puro-sh-NC for 72 h. Stable cell lines were chosen with 0.5 μg/ml puromycin and 250 μg/ml G418 for one week.

### Cell proliferation and colony formation assays

The impact of MNX1-AS1 on proliferation assay was evaluated using the Cell Counting Assay kit (CCK8, Sigma), based on manufacturer’s guidelines. Transfected cells were seeded in 96-well plates (5x10^3^ cells/well) for 24, 48 or 72 h. Next, CCK8 solution was introduced followed by a 4-h incubation. Absorbance was examined at 450 nm with a Microplate Reader (Bio-Rad, Hercules, CA, USA).

For colony formation, 1,000 plasmid incorporated cells were grown in 6-well plates over 2 weeks. Then cells were PBS-washed Twice, fixed in methanol for 15 min, and dyed with 0.1% crystal violet for 15 min at room temperature. The clones were quantified using Image J.

### Cell migration and invasion assays

Wound healing and transwell chamber assays were carried out to assess migration and invasion properties, as we previously described (9). For wound healing assay, 2 × 10^5^ transfected cells were plated in 12-well plates and allowed to grow till confluency. Next, a sterile pipette tip was employed to introduce a wound on the cell surface, before incubation in serum-free medium over 24 h before imaging at 0 and 24 h with an inverted microscope (Leica Microsystems, Inc., Buffalo Grove, IL, USA). For transwell invasion assay, 24-well Transwell chambers with polycarbonate filters (8-μm pores; Corning Inc.) were applied. Plasmid incorporated cells (1×10^4^ cells per well) in zero serum medium were introduced to the top chamber coated with Matrigel, and medium with 10% FBS was included in the bottom chamber for chemoattraction. After 24-h, the migrated cells were fixed with 4% formaldehyde for 20 min and then stained with 0.1% crystal violet for 5 min. Cell invasion was quantified with an inverted microscope (Leica Microsystems, Inc.) by choosing 5 random vision field per treatment.

### Subcellular fractionation assay

The NE-PER Nuclear and Cytoplasmic Extraction Reagents (Cat no: 78833; Thermo Fisher Scientific, Waltham, MA, USA) were used to isolate the cytoplasmic and nuclear extracts from TU212 cells. The distribution of MNX1-AS1 in cytoplasm or nucleus was examined using qRT-PCR. GAPDH and U6 served as controls for the cytoplasm and nucleus, respectively.

### Luciferase reporter assay

A wild-type (WT) or mutant (MT) MNX1-AS1 fragment containing the miR-370 binding site were introduced into the pGL3-basic vector (Promega, Madison, WI, USA).For luciferase assay, TU212 cells were simultaneously incorporated with the miR-370 mimics or corresponding NC. 48 h later, luciferase reporter assay system (Promega) was applied to examine the luciferase activity.

### RNA pull-down assay

TU212 cells were incorporated with biotinylated wide-type miR-370(Bio-wt-miR-370), mutant-type miR-370 (Bio-mt-miR-370) and negative control (bio-prote-NC, GenePharma, Shanghai, China), respectively. After 48 h transfection, lysed cells were harvested and exposed to M-280 streptaviden magnetic beads (Invitrogen) based on manufacture’s guidelines. The bead-bound-MNX1-AS1 was then quantified using qRT-PCR.

### Tumor evaluation in nude mice

All animal protocols in this study were agreed upon by the Animal Research Ethics Committee of Jilin University (Changchun, China). Ten male athymic nude BALB/c mice (5–6 weeks, 18–25g) from the Laboratory Animal center of Jilin University were housed in this center. All mice received standard mouse irradiated food and tap water *ad libitum*. TU212 cells stably incorporated with sh-MNX1-AS1 or sh-NC were subcutaneously administered into flank of nude mice (Five mice in each group). Tumor volumes were quantified weekly formulas follows: tumor volume (V) = width^2^ × length × 0.5. After 28 days, all mice were sacrificed, tumors were harvested, and weighted. The tumor was paraffin-embedded to examine the cell proliferation marker Ki-67 expression with immunohistochemical (IHC) using an anti-Ki-67 antibody (Abcam, Cambridge, UK) as described previously [13]. The residual tumor tissues were sorted at −80°C until RNA extraction.

### Statistical analysis

Each experiment was repeated 3 times and analyzed with SPSS software, version 17.0 (IBM SPSS, Armonk, NY, USA). The data presented is average ± SD (standard deviation). Continuous variables were analyzed with Student’s two-tailed *t*-test (2 groups data) or one-way analysis of variance (>2 groups data). A χ2 test was used for comparison of dichotomous variables. The differences in overall survival rate was assessed using Kaplan-Meier method and analyzed with log-rank test. Pearson's correlation analysis was employed for relationship investigations. A *P* value < 0.05 was considered as significant difference.
